# Synergistic Interaction between *Boesenbergia rotunda* (L.) Mansf. Essential Oil and Cloxacillin on Methicillin-Resistant *Staphylococcus aureus* (MRSA) Inhibition

**DOI:** 10.1155/2023/3453273

**Published:** 2023-04-16

**Authors:** Chittadech Apinundecha, Yothin Teethaisong, Siriporn Suknasang, Intu-orn Ayamuang, Griangsak Eumkeb

**Affiliations:** ^1^School of Preclinical Sciences, Institute of Science, Suranaree University of Technology, Nakhon Ratchasima 30000, Thailand; ^2^School of Biology, Institute of Science, Suranaree University of Technology, Nakhon Ratchasima 30000, Thailand; ^3^Faculty of Allied Health Sciences, Burapha University, Chon Buri 20131, Thailand; ^4^Research Unit for Sensor Innovation (RUSI), Burapha University, Chonburi 20131, Thailand

## Abstract

Currently, antibiotic resistance is widespread among bacteria. This problem requires greater awareness because bacterial resistance increases, reducing antibiotic use effectiveness. Consequently, new alternative treatments are needed because the treatment options for these bacteria are limited. This work aims to determine the synergistic interaction and mechanism of action of *Boesenbergia rotunda* essential oil (BREO) against methicillin-resistant *Staphylococcus aureus* (MRSA). Gas chromatography-mass spectrometry identified 24 BREO chemicals (GC-MS). The main components of BREO were *β*-ocimene (36.73%), trans-geraniol (25.29%), camphor (14.98%), and eucalyptol (8.99%). BREO and CLX inhibited MRSA DMST 20649, 20651, and 20652 with a minimum inhibitory concentration (MIC) of 4 mg/mL and 512 *µ*g/mL, respectively. The checkerboard method and the time-kill assay revealed synergy between BREO and CLX with fractional inhibitory concentration (FIC) <0.5 and log reduction >2log10 CFU/mL at 24 hours compared to the most effective chemical. BREO inhibited biofilm formation and increased membrane permeability. Exposure alone to BREO or in combination with CLX inhibited biofilm formation and increased cytoplasmic membrane (CM) permeability. The scanning electron microscopy (SEM) and transmission electron microscopy (TEM) results revealed that alterations in the cell walls, cytoplasmic membrane, and leakage of intracellular components of MRSA DMST 20651 after treatment with BREO alone and in combination with CLX were observed. These results indicate that BREO synergizes and could reverse the antibacterial activity of CLX against MRSA strains. The synergy of BREO may lead to novel drug combinations that increase the effectiveness of antibiotics against MRSA.

## 1. Introduction

Antimicrobial resistance (AMR) in bacteria has been rapidly increasing worldwide through various resistance mechanisms, resulting in the reduced antibacterial capability of conventional antibiotics to inhibit the growth of these resistant bacteria [1]. The high incidences have created health risks to patients and caregivers, and they have posed huge healthcare burdens globally. Patients with antibiotic-resistant infections have high medical expenses, extended hospital stays, and a high mortality rate compared to infections caused by susceptible bacteria [2]. The possible causes of AMR include excessive antibiotic use in humans and animals, lack of sanitation and hygiene, and discharge of antimicrobial residues toward the environment through fertilizer and animal waste [3].

Methicillin-resistant *Staphylococcus aureus* (MRSA) is a strain of *Staphylococcus aureus*, Gram-positive commensal bacteria that have the potential to develop resistance to several subclasses of *β*-lactams such as penicillins, cephalosporins, monobactams, and carbapenems. Furthermore, MRSA is resistant to other antibiotics, including fosfomycin, daptomycin, linezolid, chloramphenicol, gentamicin, tetracycline, fusidic acid, ciprofloxacin, and rifampicin. Correspondingly, this pathogen may cause various infectious diseases, such as bacteremia, pneumonia, osteomyelitis, prosthetic joint infection, and skin infection [4].

Methicillin resistance in MRSA is often associated with the PBP2a protein encoded by the *mec*A gene, resulting in the deletion and insertion of the *mec* element on the bacterial chromosome [5]. In addition, PBP2a facilitates cell wall synthesis while exposed to *β*-lactams due to poor *β*-lactam binding activity [6].

MRSA may produce biofilms on the surface of their habitats to protect themselves and survive in the environment. Biofilm is also one of the crucial protection mechanisms of bacteria that can disrupt or prevent the mechanisms of action of some antibacterial agents [7].

To cope with AMR in MRSA, which is resistant to several drugs, antimicrobials derived from plants are one of the treatment options due to the mechanism of action of secondary metabolites produced by plants to defend themselves against pathogens such as bacteria, fungi, and pests [8].

Essential oils are considered an interesting source of coping with these bacteria as they contain several bioactive constituents. Previous studies [9, 10] reported that some essential oils exhibited various pharmacological properties, including antibacterial, antifungal, and anti-inflammatory activity.

*Boesenbergia rotunda* (syn. *Kaempferia pandurata* Roxb or *Boesenbergia pandurata* Roxb), locally referred to in Thai as “Krachai or Krachai-Dang” and referred to in English as fingerroot, has been used as the traditional medicine in Southeast Asia due to its pharmacological properties, such as antimicrobial activities, biofilm inhibition, and antioxidant, antifungal, and anticancer activities [11]. Furthermore, this plant has also been used to combat drug-resistant bacteria, especially in the staphylococci group described by Teethaisong et al. [12].

Recently, combining conventional antibiotics with medicinal plant chemicals has become a popular strategy for reversing the antibacterial activity of failed antibiotics to treat antibiotic-resistant infections via drug interaction, which involves the effect of multiple antibacterial mechanisms. These strategies might prevent bacteria from developing novel resistance mechanisms, minimize antibiotic use while maintaining current antibiotic classes for therapeutic benefit, and mitigate undesirable effects [13].

Although there are many reports on the antimicrobial activity and synergistic interaction of *B. rotunda* against MRSA, little is available on the antimicrobial activity and synergistic interaction of the essential oil of this plant, either taken alone or in combination with conventional antibiotics, against MRSA. Therefore, this study aimed to investigate the antibacterial activity, synergistic interaction, and some mechanisms of action of BREO. Furthermore, this investigation might provide information on the therapeutic potential of BREO on MRSA inhibition, whether taken alone or in combination with conventional antibiotics such as cloxacillin.

## 2. Methods

### 2.1. Bacterial Strains and Antibacterial Agents

The Department of Medical Sciences provided MRSA isolates, including MRSA DMST 20649, 20651, and 20652. In addition, *S. aureus* ATCC 29213 was acquired from the American Type Culture Collection (ATCC) and used as the quality control strain. Sigma-Aldrich provided all antibiotics employed in this experiment, including cloxacillin (CLX) and nisin (NIS).

### 2.2. Plant Specimen and Essential Oil Preparation

*B. rotunda* rhizomes were obtained at the Suranakhon local market in the Mueang district of Nakhon Ratchasima province, Thailand. Dr. Santi Wattana from Suranaree University of Technology, Thailand, identified and verified the plant specimen. The Forest Herbarium of Thailand deposited a voucher specimen (BKF No. 192160). In this experiment, hydrodistillation was performed to extract the essential oils using a Clevenger-type apparatus [14]. 200 g of dried *B. rotunda* rhizomes was extracted by hydrodistillation of 500 mL of distilled water for 4 hours. The essential oil was dehydrated with anhydrous sodium sulfate and kept at 4°C.

### 2.3. Chemical Constituents of the Essential Oil

The constituent of BREO was determined using gas chromatography-mass spectrometry (GC-MS) following the approach described by Adams [15] with minor modifications. The essential oil was analyzed using a Bruker 450 gas chromatograph attached to a Bruker 320 mass-selective detector with the Rtx-5MS fused silica capillary column (30 m length × 0.25 mm diameter x 0.25 *µ*m film thickness). The column oven temperature was set at 40°C for 2 minutes, increased to 220°C at 30°C/min, and held at 220°C for 3 minutes. Helium was chosen as the carrier gas and injected at 1 L. Identifying the composition of this oil requires comparing its retention time to that of standard chemicals.

### 2.4. Minimum Inhibitory Concentration (MIC)

The MIC for BREO and CLX was determined following the conditions of the Clinical Laboratory Standards Institute protocol [16]. In brief, cloxacillin was prepared, and BREO was dissolved with 5% DMSO. CLX and BREO were serially diluted by a factor of 2 in the 96-well microplate containing cation-adjusted Mueller–Hinton broth (CAMHB). After 18 hours of incubation, the quantity of MRSA strains was adjusted by measuring the optical density (OD), and 10^8^ CFU/mL was obtained and diluted with normal saline to a 5 × 10^6^ CFU/mL, and 20 mL of inoculum was added to the well which included BREO or CLX and CAMHB resulting in a final concentration of 5 × 10^5^ CFU/mL and final volume of 200 *µ*L. As negative controls, wells free of antibacterial agents and bacteria were employed. The 96-well microplate was incubated at 37°C for 18 hours. The MIC value was determined as the lowest concentration that exhibited no turbidity. The MICs of antimicrobial agents were evaluated and compared to the CLSI guideline for drug resistance interpretation.

### 2.5. Checkerboard Method

The checkerboard method was carried out to determine the synergistic interaction between BREO and CLX, as previously described by Odds [17]. In the same manner as the MIC determination, BREO and CLX were prepared, and their combinatorial effect was evaluated by combining them at 37°C for 18 hours. The fractional inhibitory concentration (FIC) was determined by combining the concentrations of each antibacterial agent that inhibited the growth of the observed bacteria. The following formula was used to calculate and interpret the FIC index.

(1) $$\begin{array}{c} FIC\;index=FICA+FICB=\frac{\text{Conc}.\text{ of }A\text{ in MICs of }A+B}{\text{MIC of }A\text{ alone}}+\frac{\text{Conc}.\text{ of }B\text{ in MICs of }A+B}{\text{MIC of }B\text{ alone}}\text{.} \end{array}$$

The FICI can be described as synergism, no interaction, and antagonism whenever the FIC value is ≤0.5, >0.5–4.0, and >4.0, respectively.

### 2.6. Time-Kill Assays

Time-kill assays were performed to illustrate antibacterial and synergistic activity against MRSA 20651, with minor adjustments to the procedure described by Teethaisong et al. [12]. In brief, the inoculum (5 × 10^6^ CFU/mL) was exposed to BREO, CLX alone, or in combination for 6 exposure periods (0, 2, 4, 6, 8, and 24 hours). 0.1 mL of aliquots from each treatment interval was diluted with 0.9 mL of normal saline. 10 *µ*L of each dilution was dropped on Mueller–Hinton agar (MHA). After 18 hours of incubation at 37°C, the nutrient plate containing 3–50 colonies were chosen to count using the surface drop method or the Miles and Misra method, which was tested to be as accurate and time-saving as described by Hedges et al. [18, 19]. Then, time-kill curves were plotted. CFU/mL was calculated using the following formula:

(2) $$\begin{array}{c} \frac{CFC}{mL}=\text{average number of colonies in each dilution}\times 100\times \text{dilution factor}. \end{array}$$

At 24 hours, the synergistic interaction was considered as ≥2 log_10_ reductions in CFU/mL of the combined agent-treated group compared to the single most effective agent-treated group [20]. In addition, the bactericidal effect was described as a reduction ≥3log_10_ CFU/mL, and the bacteriostatic effect was determined to be a decrease less than 3log_10_ CFU/mL of each treatment group at 24 hours compared to the starting inoculum [21].

### 2.7. Cytoplasmic Membrane (CM) Permeability

This experiment was performed as previously described by Siriwong et al. [22] with a slight modification. The CM damage was determined by measuring the intensity of the OD_260_-absorbing materials using a UV-VIS spectrophotometer. After incubation for 18 hours, the MRSA was collected and adjusted to a concentration of 5 × 10^6^ CFU/mL in normal saline. Modified cultures (5 mL) were added to 45 mL of CAMHB supplemented with BREO, CLX alone at half-MIC, or BREO plus CLX at FIC concentrations. As a negative control, a flask without an antibacterial agent was utilized. Nisin was applied as a positive control to increase CM permeability in this experiment because it can damage the cytoplasmic membranes of Gram-positive bacteria. These bacterial cultures were incubated at 37°C in a shaking incubator. The CM permeability was determined at 0, 1, 2, 3, and 4 hours. In addition, the OD_260_ intensity of UV-absorbing materials leaked from the cells was evaluated in the supernatant, as described by Paul et al. [23]. All tests were done in triplicate with a Varian Cary 1E UV/VIS spectrophotometer.

### 2.8. Biofilm Formation Inhibition

Biofilms are formed when a bacterial colony generates polysaccharides, proteins, nucleic acids, and lipids. Bacteria are held together by the extracellular matrix, which creates a three-dimensional film-like structure. Biofilm formation is an antibiotic resistance mechanism that contributes to persistent infections by decreasing the penetration of the drug through these films. Consequently, the inhibitory effect of BREO on biofilm growth was evaluated using the methodology described by He et al. [24] with some modifications. First, the bacterial culture was counted to 5 × 10^6^ CFU/mL in saline solution after incubation for 18 hours. In 96-well microtiter plates, 20 *µ*L of bacterial inoculum was added to 180 *µ*L of CAMHB supplemented with 0.2% glucose and a half-MIC or FIC of BREO, depending on whether it was used alone or in combination with CLX. These solutions were incubated at 37°C for 48 hours. Then, the bacterial medium was removed, and adhering cells on the surface of each well were rinsed with distilled water and stained for 30 minutes with a crystal violet solution containing 0.4% (w/v) crystal violet. After dyeing, the crystal violet solution was washed with distilled water. After that, air-dried adherent cells stained with crystal violet were washed in 100% ethanol in each well. A microplate reader set to 595 nm was used to determine the optical density of the solution in each well. Antibiofilm formation was evaluated through the percentage of inhibition calculated following the formula presented in the study by Gómez-Sequeda et al. [25].

(3) $$\begin{array}{c} \%\text{ inhibition}=\frac{\text{OD negative control}-\text{OD treatment group}}{\text{OD negative control}}\times 100\text{.} \end{array}$$

### 2.9. Scanning Electron Microscopy (SEM)

The SEM sample preparation procedure was performed following the method of Hartmann et al. [26] with slight adjustments. In brief, MRSA DMST 20651 strain was cultured in CAMHB at 37°C for 18 hours and then adjusted to a final concentration of 5 × 10^5^ CFU/mL. This strain was treated with CLX and BREO alone at half-MIC and CLX plus BREO at FIC at 37°C for 4 hours. The positive control was chosen and incubated in an antibiotic-free medium. Next, this strain was fixed with 2% glutaraldehyde in 0.15 M sodium phosphate buffer (pH 7.2), rinsed, and resuspended in distilled water. Then, samples were incubated with 0.5% osmium tetroxide (OsO_4_) for 2 hours. The samples were dehydrated using a graded acetone solution (20%, 40%, 60%, 80%, and 100%,respectively), dried in the air, mounted on a carbon stub, and sputtered with gold. Finally, images of the cell morphology of these samples were captured using a scanning electron microscope.

### 2.10. Transmission Electron Microscopy (TEM)

The TEM was used to evaluate the structural damage of bacteria produced by BREO or BREO plus CLX. The procedure for sample preparation was performed following the method of Richards et al. [27] with minor modifications. In brief, after 18 hours of incubation, the final concentration of bacterial suspension was adjusted to 5 × 10^5^ CFU/mL, then incubated for 3 hours at 37°C, and shaken at 110 rpm in a shaking incubator. This suspension was centrifuged at 6000 × *g* for 15 minutes at 4°C, the supernatant was removed, and the pellet was fixed for 12 hours in 2.5% glutaraldehyde-containing 0.1 M phosphate buffer (pH: 7.2). The samples were rinsed twice in 0.1% phosphate buffer and incubated for 2 hours in 1% OsO_4_ at room temperature. This sample was dehydrated for 15 minutes using a graded concentration of acetone solution (20%, 40%, 60%, 80%, and 100%, respectively). The epoxy resin was used to embed these samples. Afterward, these samples were counterstained for 3 minutes with 2% (w/v) uranyl acetate and 2 minutes with 0.25% (w/v) lead citrate. The specimens were then observed and photographed using a 80kV electron microscope. Note that the bacteria growing without CLX served as the control treatment. Cell area was computed to examine the impact of BREO alone and combined with CLX on cell size by multiplying cell width by cell length in TEM images (nm^2^).

### 2.11. Statistical Analysis

The statistical method was performed using IBM SPSS Statistics 22. The data were represented by mean ± standard error of the mean (SEM). The significant differences in CM permeability, biofilm density, and cell area between treated groups were determined using a one-way analysis of variance (ANOVA). Post hoc Tukey's HSD (honestly significant difference) test was compared at a *P* value<0.01.

## 3. Results

### 3.1. Gas Chromatography-Mass Spectrometry (GC-MS)

The chemical identification of essential oils was determined by comparing their retention times and mass spectra to a database of reference compounds. There were 24 compounds found in BREO, representing 100% of the overall constitution. The main constituents of BREO were *β*-ocimene (36.73%), trans-geraniol (25.29%), camphor (14.98%), and eucalyptol (8.99%) (Table 1).

### 3.2. Minimum Inhibitory Concentration (MIC)

The result of MIC determination demonstrated that BREO inhibited MRSA DMST 20649, 20651, and 20652 at a MIC of 4 mg/mL. In *S. aureus* ATCC 29213, the BREO showed a MIC of 2 mg/mL for this strain. CLX resistance was observed in MRSA DMST 20649, 20651, and 20652 strains with MIC of 512 *µ*g/mL. *S. aureus* ATCC 29213 was sensitive to CLX with MIC of 0.125 *µ*g/mL (Table 2).

### 3.3. Checkerboard Method

The synergistic interaction between BREO and CLX was found in MRSA DMST 20649, 20651, and 20652 with an FIC index<0.5. The concentration of BREO and CLX in the combined test was much lower than that of the single chemical concentration (Table 3).

### 3.4. Time-Kill Assay

The inhibitory action of BREO alone and in combination with CLX against MRSA DMST 20651 is shown in Figure 1. The findings demonstrated that the growth of the untreated control group was normal. Cell viability after exposure to half-MIC of CLX (256 *µ*g/mL) and BREO (2 mg/mL) revealed growth reduction during the first 6 hours of incubation, after which bacteria started to multiply. After being treated with BREO (1 mg/mL) plus CLX (16 *µ*g/mL), the growth of the bacteria displayed a steady decrease in viable cell count after the first 4 hours of incubation until 24 hours. The group treated with the combined chemical revealed >2log_10_ reduction in viable cells compared to the single most effective group (BREO-treated group). Therefore, this combined chemical exhibited a synergistic interaction against MRSA DMST 20651. Additionally, the combined group also exhibited a <3log_10_ decrease in CFU at 24 hours relative to the initial CFU, indicating a bacteriostatic effect.

### 3.5. Cytoplasmic Membrane (CM) Permeability

Figure 2 shows the findings of CM permeability tests. Compared to the control group, the CLX-treated group did not exhibit any OD_260_-absorbing material leakage after 1 hour of treatment (*p* > 0.01). OD_260_ of cells treated with BREO, nisin, or BREO plus CLX considerably increased compared to cells treated with CLX alone or a control (*p* < 0.01). There was no statistically significant difference throughout the experiment between cells treated with BREO and those treated with BREO plus CLX (*p* > 0.01), except for the 3 hours in which BREO plus CLX exhibited significantly higher cytoplasmic membrane permeability.

### 3.6. Biofilm Formation Inhibition

A typical quantitative biofilm result exhibited that CLX and BREO, either alone or in combination, prevented the development of biofilms against MRSA 20651, as seen in Figure 3. After 48 h of treatment, MRSA 20651 cultured without antibacterial drug exhibited the highest biofilm biomass. The percentage inhibition of the BREO-treated group, the CLX-treated group, and the combined group was 67.58 ± 0.67, 72.61 ± 0.61, and 80.25 ± 0.60, respectively. All treated groups substantially reduced the biofilm of MRSA 20651 compared to the control group (*p* < 0.01). CLX also showed more significant biofilm inhibition activity than BREO (*p* < 0.01). Besides, the combination of BREO (1 mg/mL) and CLX (16 *µ*g/mL) also revealed the highest biofilm inhibition activity compared to BREO and CLX alone (*p* < 0.01).

### 3.7. Scanning Electron Microscopy (SEM)

MRSA DMST 20651 cells were treated with BREO, CLX, and BREO plus CLX. Untreated cells displayed a cluster of berry-shaped cells with smooth cell surfaces (Figure 4(a)). After treatment with 256 *µ*g/mL of CLX, most damaged cells revealed dents (squared arrow). Additionally, some cells with a rough surface (dotted arrow) and others with withered cells (arrow) were observed (Figure 4(b)). These cells, after exposure to 2 mg/mL of BREO, displayed clefts (dotted arrow), a bleb-like structure on the cell surface (squared arrow), and cell lysis with large debris (arrow) (Figure 4(c)). Dents (arrows), clefts (squared arrows), bleb-like structures on the cell surface (dotted arrows), and significant cell lysis (rectangle arrows) were displayed in cells treated with 1 mg/mL of BREO and 16 *µ*g/mL of CLX (Figure 4(d)).

### 3.8. Transmission Electron Microscopy (TEM)

TEM was applied to assess the cell damage caused by exposure to BREO, CLX, and BREO plus CLX. The MRSA DMST 20651 cells were investigated by TEM treated with BREO (2 mg/mL), CLX (256 *µ*g/mL), BREO (1 mg/mL) plus CLX (16 *µ*g/mL), and untreated cells. In addition, the effect of such compounds on the cell sizes of each group was compared.  Figure 5(a) illustrates the structure of untreated, antibacterial-free control. These cells were allowed to grow normally. Untreated cells have a spherical and clear appearance. The cytoplasmic membrane and cell wall were distinguishable from cells treated with other treatment groups. After exposure to CLX at a concentration of 256 *µ*g/mL, the cell wall of the MRSA 20651 strain exhibited morphological changes between the cell wall and the cytoplasmic membrane (arrow) (Figure 5(b)).  Figure 5(c) displays cells treated with 2 mg/mL of BREO. The hairpin-like structure of the cytoplasmic membrane indicated the presence of alterations of the cytoplasmic membrane (arrow). Therefore, these results suggest that BREO suppresses MRSA 20651 by interacting with the cytoplasmic membrane. After exposure to the combination of 1 mg/mL of BREO and 16 *µ*g/mL of CLX, the cell wall in this group was peeled off (arrow). Additionally, the cytoplasmic membrane (squared arrow) and intracellular components (dotted arrow) were lost after exposure to this combination (Figure 5(d)). As shown in Figure 6, the cell areas of the untreated control (CTR) and cells treated with BREO, CLX, and BREO plus CLX were calculated to determine the impact of each treatment on cell size. The untreated control had a cell area of approximately 6.18 × 10^5^ ± 3.51 × 10^4^ nm^2^. This finding did not reveal statistically significant variation in cell area between the CTR, CLX-treated (5.85 × 10^5^ ± 1.31 × 10^4^ nm^2^), and BREO-treated groups (5.20 × 10^5^ ± 1.07 × 10^4^ nm^2^) (*p* > 0.01). Additionally, only the CLX plus BREO (4.34 × 10^5^ ± 1.76 × 10^4^ nm^2^) group revealed a significant reduction in cell area compared to the untreated control group (*p* < 0.01). However, this combination did not show significant differences in cell area from the BREO-treated group. These findings demonstrate that exposure of MRSA DMST 20651 to BREO plus CLX can reduce cell area.

## 4. Discussion

Due to their accessibility, affordability, and safety, medicinal plant-derived chemicals are recognized as fascinating sources of antimicrobial agents against various infections [28]. In recent years, people have tended to rely on herbal plants as sources of novel therapeutics, including for treating bacterial infections. This approach provides the way for the development of modern medicine.

*B. rotunda* is also an exciting alternative to treat antibiotic-resistant bacterial infections. This plant has shown a synergistic interaction with various antibiotics through various antibacterial mechanisms derived from secondary metabolites such as alkaloids, flavonoids, and essential oils [11, 12]. Since the evaluation of *B. rotunda*, the effectiveness of essential oils, both as single and combined therapies, identifying the main active constituent and the mechanism of action still needs to be investigated. In this work, the constituents of BREO were evaluated using the GC-MS technique. The findings found that the main components of BREO were *β*-ocimene, trans-geraniol, camphor, and eucalyptol.

Chi et al. [29] reported that essential oils extracted from citrus leaves, including *Citrus sinensis*, *Citrus grandis*, and *Citrus aurantifolia* that contained *β*-ocimene as a major constituent, demonstrated antibacterial activity against *S. aureus*, *Bacillus cereus*, and *Salmonella typhimurium* with inhibition zones and MIC values ranging from 20.1 ± 0.1 to 24.3 ± 0.1 mm and 5.25 to 21 mg/mL, respectively. Due to the antibacterial potential against *S. aureus*, *C. sinensis*, with the highest *β*-ocimene content compared to the other two species, revealed the highest inhibition effect on MRSA with a zone of 23.2 ± 0.2 mm and the lowest MIC value at a concentration of 5.25 mg/mL. Furthermore, Jaradat et al. [30] found that *Thymus bovei* essential oil containing trans-geraniol exhibited antibacterial activity against *S. aureus* and *Escherichia coli*, with MIC values of 0.25 mg/mL and 0.5 mg/mL, respectively. Camphor oil extracted from *Cinnamomum camphora* had antibacterial activity against *Streptococcus* mutants and *Enterococcus faecalis*, Gram-positive bacteria [31]. Similarly, Lopes-Lutz et al. [32] demonstrated that camphor-enriched essential oils extracted from plants in the genus *Artemisia* had antibacterial action against *S. aureus*, with inhibition zones between 10 ± 0.0 and 25 ± 1.4 mm, compared to 8 ± 0.5 and 18 ± 1.0 mm for methicillin and vancomycin, respectively. These oils were also found to have antifungal efficacy with an inhibition zone ranging from 15 ± 1.4 to 40 ± 2.1 mm against *Microsporum canis*, while amphotericin B exhibited an inhibition zone of 19 ± 1.0 mm. Hamad Al-Mijalli et al. [33] provided the details of *Lavandula multifida* essential oils (LMEOs) containing eucalyptol inhibiting the growth of *S. aureus*, *Listeria monocytogenes*, *Bacillus subtilis*, and *E. coli*, with MIC values ranging from 0.78 to 1.56 mg/mL. Regarding the antibacterial activity determined in this study, the MIC value of BREO was 4 mg/mL. This antibacterial action against MRSA strains may be attributable to the activity of *β*-ocimene, trans-geraniol, camphor, and eucalyptol.

Although using BREO or CLX monotherapy to inhibit MRSA had low activity, the combination of BREO and CLX showed higher antibacterial action from the synergistic interaction. This finding is in accordance with a previous investigation that the combination of geraniol and norfloxacin had a synergistic interaction (FIC <0.5) against *B. cereus* and *S. aureus* isolates; besides, the combination of geraniol and chloramphenicol synergistically inhibited *E. coli*, *Klebsiella pneumoniae*, *Proteus mirabilis*, and *P. aeruginosa* [34]. Similar to a study by Bekka-Hadji et al. [35], *Artemisia herba-alba* essential oil containing camphor exhibited a synergistic interaction with cephalosporins against *S. aureus*. Requena et al. [36] reported that the synergistic interaction occurred when 1 mg/mL of eucalyptol was combined with thymol and cinnamaldehyde at a concentration of 0.05 and 0.1 mg/mL, respectively, against *Listeria innocua*. Our work determined the synergistic interaction using a checkerboard assay, and FIC <0.5 was found, which ODD theory interpreted as a synergistic interaction [17]. In the time-kill experiment, the concentration of each chemical was selected depending on the MIC value. The half-MIC concentrations of BREO and CLX were chosen because these concentrations did not inhibit bacteria growth at around 24 hours of incubation. Usually, the synergistic interaction of the combined chemical can inhibit bacterial growth at doses of each chemical that are less than half the MIC of a single chemical. The finding of this assay demonstrates that the combined drug reduces the growth of MRSA DMST 20651 >2log_10_ CFU/mL compared to the most effective chemical (BREO) at 24 hours. This growth reduction was observed from the start and throughout 24 hours after exposure to the half-MIC of BREO and CLX. The findings of the time-kill assay support the checkerboard method that two chemicals show a synergistic interaction. This synergistic interaction may be influenced by the main constituents of BREO mentioned above. Therefore, the synergistic approach must be verified by investigating the mechanism of action of BREO and CLX, which inhibits cell wall synthesis.

According to the investigation of the mechanism of action, the concentration of chemicals was selected from those used in time-kill tests, ensuring consistency throughout all experiments, following the pattern of Siriwong et al. [22] with some modifications. Furthermore, using concentrations below the MIC value of a single chemical enables a better understanding of the mechanism of action, especially the morphological alteration observed by SEM and TEM, because these concentrations are insufficient to kill all bacteria. The mechanism of action in this work was focused on determining the synergistic interaction of BREO on the alteration of CM permeability and the antibiofilm formation activity.

Regarding the permeability of CM, Asker et al. [37] indicated that the mechanism of *β*-ocimene in the inhibition of *S. aureus* and *Pseudomonas aeruginosa* was by inhibiting the biosynthesis of lipids of these bacteria in a concentration-dependent manner. According to Tang et al. [38], the essential oil of *Amomum villosum* Lour., containing 20.94% camphor, induced increasing membrane permeability, resulting in leakage of intracellular components, especially DNA and RNA. Furthermore, it was proposed that the mechanism of action of geraniol in inhibiting several pathogens was by adhering and interacting with the membrane lipid of the microbe, resulting in increased membrane permeability [34]. This work determined the permeability of CM by measuring the intensity of OD_260_, which was explicitly related to the number of intracellular components that leaked out of the cell, such as DNA and RNA. The result demonstrated that the BREO-treated and combined groups increased the CM permeability more than the untreated control and CLX-treated groups. Furthermore, at 4 hours of incubation, the permeability of CM after exposure to the combined drug was not significantly different from that of nisin, which was used as a positive control in previous studies [12, 39]. These results imply that the combination of BREO and CLX could increase the permeability of bacterial CM and may be acted by the main components of BREO, such as *β*-ocimene, camphor, and trans-geraniol. The antibacterial action of nisin is well known to destroy the bacterial cell membrane. It was employed as a positive control agent for a cell membrane permeability assay in this study. Although nisin substantially increased CM permeability, it is an alternative drug for treating MRSA infection [40]. This study focused on combining BREO and CLX to reverse practically used antibiotics that have lost their antibacterial activity. Hence, using nisin in combination with BREO was not considered in this work.

For antibiofilm formation activity, geraniol and camphor exhibited antibiofilm activity by inhibiting *S. aureus* biofilm with the inhibition percentage of 86.13 ± 5.22 and 81.25 ± 1.63 after exposure to 256 *µ*g/mL of geraniol and 10 mg/mL of camphor, respectively [41, 42]. Furthermore, Vijayakumar et al. [43] found that eucalyptol showed a concentration-dependent manner for inhibition of biofilm formation of *Streptococcus pyogenes* by 89% inhibition after exposure to this chemical at a concentration of 300 *µ*g/mL. Therefore, in our work, the antibiofilm activity of BREO may be due to these compounds mentionedearlier. Adeyemo et al. [44] reported the criteria that good antibiofilm formation occurred when the percentage inhibition was more significant than 50%. These results provide evidence that CLX, BREO, and its combination demonstrate a good effective inhibition of biofilm formation with percentage inhibition of 67.58 ± 0.67, 72.61 ± 0.61, and 80.25 ± 0.60, respectively. In addition, the combined drug exhibited the highest biofilm inhibition activity compared to other groups (*p* < 0.01). Therefore, the combination with a lower concentration of each compound exhibits significantly higher antibiofilm activity than a single one with a higher concentration. This finding is consistent with previous studies that the main constituents of BREO revealed antibiofilm formation activity.

TEM and SEM analyses were performed on cells exposed to BREO, CLX, and their combinations to determine the position of action based on morphological changes. After exposure to BREO, hairpin-shaped coiling of the cytoplasmic membrane could be indicated as an alteration. CLX was responsible for cell wall deformation. However, damage to the cell wall and the cytoplasmic membrane was observed when BREO was combined with CLX. Furthermore, this combination of BREO and CLX displayed the action through several mechanisms, such as inhibition of cell wall synthesis, increased CM permeability, and antibiofilm formation activity, consistent with the purpose of the study. These findings are consistent with Teethaisong et al. [12] and Siriwong et al. [22] that synergistic interaction could occur when two chemicals with different mechanisms of action inhibit bacteria concurrently.

To fully understand BREO's antibacterial and synergistic properties, additional modes of action associated with resistance mechanisms, cytotoxicity tests, safe dosage for human and animal cells, and the total content of active constituents must be considered in a future perspective. This state of knowledge could lead to additional learning on issues relevant to the synergistic interaction of natural chemicals and conventional antibiotics. Taken together, BREO could synergistically restore the activity of CLX that failed to treat MRSA infections. This could lead to the development of novel treatment options for infections caused by multidrug-resistant MRSA.

## 5. Conclusions

In summary, BREO demonstrates an inhibitory effect on *β*-lactam-resistant staphylococci. The mechanism of action of this essential oil is most likely to act at the cytoplasmic membrane, resulting in alterations in the cytoplasmic membrane. Furthermore, another mode of action is biofilm formation inhibitory activity. The synergistic activity of BREO and CLX against MRSA DMST 20651 strains can be attributed to the reduction in biofilm production and increase in cytoplasmic membrane damage resulting in the leakage of cellular components.

## Figures and Tables

**Figure 1:** Cell viability of MRSA DMST 20651 cells after exposure to BREO and CLX, whether alone or in combination. CTR = control, CLX = CLX at 256 *µ*g/mL, BREO = BREO at 2 mg/mL, and CLX + BREO = CLX at 16 *µ*g/mL plus BREO at 1 mg/mL. The values were represented by the mean and standard error of the mean (SEM) from triplicates.

**Figure 2:** Change in quantity of OD_260_-absorbing material of MRSA DMST 20651 after treatment with BREO and CLX, whether taken alone or in combination. CTR = control, CLX = CLX at 256 *µ*g/mL, BREO = BREO at 2 mg/mL, and CLX + BREO = CLX at 16 *µ*g/mL plus BRE at 1 mg/mL. NIS = nisin at 8 *µ*g/mL. The values were represented by the mean and standard error of the mean (SEM) from triplicates. The one-way ANOVA and Tukey's HSD post hoc tests were compared between results. The different alphabetical symbols indicate a statistically significant difference between groups (*p* < 0.01).

**Figure 3:** The inhibition of MRSA 20651 biofilms was quantified after treatment with BREO, or CLX, either alone or in combination. CTR = control, CLX = CLX at 256 *µ*g/mL, BREO = BREO at 2 mg/mL, and CLX + BREO = CLX at 16 *µ*g/mL and BREO at 1 mg/mL. The values were represented by the mean and standard error of the mean (SEM) for six replicates. The one-way ANOVA and Tukey's HSD post hoc tests were compared between results. The different alphabetical symbols indicate a statistically significant difference between groups (*p* < 0.01).

**Figure 4:** MRSA DMST 20651 SEM images after incubation in CAMHB (100 nm and 20000x) (a) and after exposure to 256 *µ*g/mL of CLX (200 nm and 15000x) (b), 2 mg/mL of BREO (300 nm and 15000x) (c), and 1 mg/mL of BREO plus 16 *µ*g/mL of CLX (200 nm and 15000x) (d).

**Figure 5:** MRSA DMST 20651 TEM images after incubation in CAMHB (original: 1 *µ*m and 10000x; inset: 100 nm and 89000x) (a) and after exposure to 256 *µ*g/mL of CLX (original: 500 nm and 13000x; inset: 100 nm and 89000x) (b), 2 mg/mL of BREO (original: 1 *µ*m and 8500x; inset: 100 nm and 89000x) (c), and 1 mg/mL of BREO plus 16 *µ*g/mL of CLX (original: 500 nm and 17000x; inset: 100 nm and 89000x) (d)

**Figure 6:** The effect of BREO, CLX, and BREO plus CLX on the cell area of MRSA 20651. CTR = untreated control, BREO = *B. rotunda* essential oil at a concentration of 2 mg/mL (*n* = 6), CLX = cloxacillin at a concentration of 256 *µ*g/mL (*n* = 6), and BREO + CLX = *B. rotunda* essential oil at a concentration of 1 mg/mL and cloxacillin at a concentration of 16 *µ*g/mL (*n* = 6). The cell area was calculated by the cell width multiplied by the cell length (nm^2^). Using one-way ANOVA with Tukey's HSD, different alphabets indicate a statistically significant difference (*p* < 0.01). The data were presented as the mean and standard deviation of the mean (SEM).

**Table 1:** Chemical constituents present in *B. rotunda* essential oil.

Retention time (RT) (min)	Peak name	% area
9.502	Tricyclene	0.16
9.872	alpha-Thujene	0.01
10.164	alpha-Pinene	0.65
10.969	Camphene	4.45
12.565	beta-Pinene	0.11
13.745	beta-Myrcene	1.00
14.380	alpha-Phellandrene	0.04
15.180	alpha-Terpinene	0.05
16.113	**Eucalyptol**	**8.99**
16.877	trans-beta-Ocimene	3.92
17.783	**beta-Ocimene**	**36.73**
18.108	gamma-Terpinene	0.06
19.987	Terpinolene	0.15
21.166	beta-Linalool	1.01
23.807	**Camphor**	**14.98**
24.000	Camphene hydrate	0.36
24.665	Isoborneol	0.04
25.320	endo-Borneol	0.28
26.091	4-Terpineol	0.13
27.126	alpha-Terpineol	0.43
32.157	**trans-Geraniol**	**25.29**
32.716	alpha-Citral	0.15
39.831	Methyl cinnamate	1.01
51.294	Caryophyllene oxide	0.01
Total		100.00

The high value of chemical constituents is represented by bold values.

**Table 2:** Minimum inhibitory concentrations (MICs) of cloxacillin (CLX) and *B. rotunda* essential oil (BREO) against *S. aureus* strains.

Bacterial strains	Minimum inhibitory concentration (MIC)	
	CLX (*µ*g/mL)	BREO (mg/mL)
MRSA DMST 20649	512^*R*^	4^*ND*^
MRSA DMST 20651	512^*R*^	4^*ND*^
MRSA DMST 20652	512^*R*^	4^*ND*^
*S. aureus* ATTC 29213^*∗*^	0.125^*S*^	2^*ND*^

^*∗*^A reference strain. ^*R*^Resistant; ^*S*^susceptible; ^*ND*^no data available.

**Table 3:** Fraction inhibitory concentration (FIC) index of cloxacillin (CLX) plus *B. rotunda* essential oil (BREO) against *S. aureus* strains.

Bacterial strains	MIC(a)		MIC(c)		FIC		FICI
	BREO (mg/mL)	CLX (*µ*g/mL)	BREO (mg/mL)	CLX (*µ*g/mL)	BREO	CLX	
MRSA DMST 20649	4^*ND*^	512*^R^*	1^*ND*^	16*^R^*	0.25	0.03	0.28^*∗*^
MRSA DMST 20651	4^*ND*^	512*^R^*	1^*ND*^	16*^R^*	0.25	0.03	0.28^*∗*^
MRSA DMST 20652	4^*ND*^	512*^R^*	1^*ND*^	32*^R^*	0.25	0.06	0.31^*∗*^

^*∗*^Synergistic interaction (FIC index ≤0.5). FICI = FIC index; MIC(a) = MIC value of chemical alone; MIC(c) = MIC value of chemical in combined drug. ^*R*^Resistant; ^*S*^susceptible; ^*ND*^no data available.

## Data Availability

The data used to support the findings of this study are included within the article.
